The article "A Novel Virtual Reality Training Strategy for Poststroke Patients: A Randomized Clinical Trial" was published in 2021. Journal: J Healthc Eng.

# A Novel Virtual Reality Training Strategy for Poststroke Patients: A Randomized Clinical Trial

**DOI:** 10.1155/2021/6598726

**Published:** 2021-11-18

**Authors:** Naveed Anwar, Hossein Karimi, Ashfaq Ahmad, Nazia Mumtaz, Ghulam Saqulain, Syed Amir Gilani

**Affiliations:** ^1^Physical Therapy Department, University of Lahore, Lahore 42000, Pakistan; ^2^Riphah College of Rehabilitation & Allied Health Sciences, Riphah International University, Lahore 42000, Pakistan; ^3^Faculty of Allied Health Sciences, Riphah International University, Lahore 42000, Pakistan; ^4^Department of Otorhinolaryngology, Capital Hospital PGMI, Islamabad 44000, Pakistan

## Abstract

Stroke patients suffer impairments including sensory, motor, visual, and cognitive areas, as well as gait and balance manifestations making activities of daily living difficult. In such conditions, virtual reality training can be a potential rehabilitation tool in comparison to conventional physical therapy to cater to the burden of this disability; hence, this randomized clinical trial compared the effects of virtual reality training and conventional physical therapy on balance and lower extremity function in stroke patients. The sample of 68 poststroke participants from Kanaan Physical Therapy and Spine Clinic, Lahore, Pakistan, were divided into *N* = 34 cases each using the lottery method with one group given virtual reality training and the other received conventional physical therapy. Each group received 60 minutes intervention, 3 days per week for 6 weeks. The Berg balance scale and the Fugl-Meyer assessment-lower extremity scale were employed for data collection preintervention, immediate postintervention, and 6 weeks postintervention. The statistically significant differences between virtual reality and conventional physical therapy groups for the Berg Balance score (*p* < 0.001), Fugl-Meyer assessment (FMA)-lower extremity domains of FMA-motor function (*p* < 0.001), FMA-joint pain, and joint range (*p* < 0.001); however, there is no significant difference (*p*=0.202) for time vs. group interaction and significant (*p* < 0.001) for the time main effect for FMA sensation. Hence, virtual reality training is more effective to restore balance and lower extremity function compared to conventional physical therapy in stroke patients. The results of the study have significant implications for the clinicians with better case management enhancing quality of life of patients along with the dearth of local literature, thus providing base for future research from a developing country's perspective.

## 1. Introduction

Stroke or cerebrovascular accidents (CVA) are considered as the leading cause of disability globally with more youth being affected in developing countries [1]; however, there is equal gender prevalence marring quality of life (Qol) at every level. Stroke has a global lifetime risk of 24.9% estimated in 2016 and extrapolated estimates by 2030 with 4% of population having a stroke event during the lifetime mounting medical costs to $ 183.13 billion [2]. The patients with stroke may have a wide variety of impairments in motor, sensory, visual, and cognitive areas including gait deficits and balance-related manifestations [3]. Hence, they experience restrictions to participate in activities of daily living (ADLs) and compromising the Qol. In addition to improved preventive and acute care facilities, neurorehabilitation is a ray of hope to cater to the burden of disability among this population [1, 4].

The article "A Novel Virtual Reality Training Strategy for Poststroke Patients: A Randomized Clinical Trial" was published in 2021. Journal: J Healthc Eng.

Looking at the prospects of mobility, conventional physical therapy (PT) is employed in lower limb rehabilitation including exercises and certain balance techniques. A study by de Rooij et al. involving community dwellers examined by virtual reality (VR) gait training and non-VR gait training containing conventional functional gait exercises and treadmill training was seen as effective in stroke patients; however, VR training showed better results compared to conventional therapeutic interventions [5].

Researchers have elaborated on the advancement of the neuroplastic changes connected with poststroke motor impairment and the inherent repair mechanisms [6]. An important role has been determined with PT focusing on the sensory input reflecting improvement in the neuroplasticity with sensory and motor learning [7]. When the patient observes his/her movements, the plasticity changes that depend on the use of sensory areas belonging to the mirror neuron system are strengthened. This exemplifies, among other factors, the improvements the Wii can provide in such patients. Moreover, this feedback could lead to a strengthening of the learning mechanisms of different motor and sensory activities that would ultimately improve quality of life [8].

The poststroke balance rehabilitation using different therapies is in use, and further research has been proposed [9]. A local study by Saleem has also emphasized on the need of clinical trials comparing VR gaming with conventional rehabilitation for stroke patients in Pakistan [10].

VR has achieved a greater attention in recent times, and it is an adjuvant rehabilitation method capable of producing neuroplasticity with the help of visual, sensory, as well by evoking cognitive interactions at the intercortical level. Its application by robotics has shown to restore the lower limb function by inducing neuroplasticity [11]. A number of randomized clinical trials have appraised the Nintendo Wii-based rehabilitation of stroke patients especially the balance. The research by Cho et al. worked on the balance training of stroke patients by using Nintendo Wii gaming. The results showed significant improvement of dynamic balance [12]. In contrast, another study conducted by Fritz et al. [13] revealed only slight improvement in balance in the Nintendo Wii group as compared to the control group. While VR has shown improvement in motor function and functional capacity in Nintendo Wii®, electronic game for the stroke survivors to improve sensorimotor rehabilitation [14] has shown to have higher impact on improvement of balance and fall prevention than conventional PT [15]. It has also been noted to be cost-effective therapeutic intervention [16] and hence needs to be considered for a developing country like Pakistan.

The article "A Novel Virtual Reality Training Strategy for Poststroke Patients: A Randomized Clinical Trial" was published in 2021. Journal: J Healthc Eng.

Stroke is 5–10 times more prevalent in certain countries including Pakistan compared to the west, with South Asia sharing 20% of the world's population and shouldering the highest burden of cardiovascular disease. This is marred with high incidence of stroke in the middle-aged group with 1/3^rd^ strokes occurring in those <45 years age accompanied with more prevalent risk factors especially nontraditional ones including the use of local drugs like naswar, smoking of pipe, and chewing betel leaf (paan) and higher incidence of diseases like rheumatic heart disease and liver diseases [17–19]. This is also associated with higher prevalence of hypertension at younger age with increased frequency of lacunar infarcts among ischemic stroke, a subtype of stroke in Pakistan that differs from Western literature as reported [20–22]. With the rate of prevalence and the fact is that Pakistan, harbouring a young population of 63% aged between 15 and 33 years, could be facing a grave health peril [23]. Hence, the need to focus on younger age groups for research seems inevitable. Good posture and adequate balance maintenance are essential prerequisites for performing active ADLs and therefore should be targeted in rehabilitation interventions [12].

Thus keeping in view the unique position of stroke in Pakistan with epidemiological and the clinical dissimilarities with the Western literature, especially due to the involvement of the younger population and the cost-effectiveness of VR, there is a need to establish the fact that neurorehabilitation using virtual therapy to improve the balance and gait of poststroke cases is a better option compared to conventional therapies, and in this connection, there is need of randomized clinical trials (RCT) for evaluation of impact of VR on balance [24].

The article "A Novel Virtual Reality Training Strategy for Poststroke Patients: A Randomized Clinical Trial" was published in 2021. Journal: J Healthc Eng.

Hence, this study was conducted to compare the effects of VR training and routine PT on balance and lower extremity function in stroke patients, with the hypothesis that VR training is better than conventional PT for balance and lower extremity function restoration in 40–60 years old stroke patients.

## 2. Materials and Methods

This single (assessor) blinded randomized clinical trial recruited diagnosed stroke patients using convenience sampling from Kanaan Physiotherapy and Spine Clinic, Lahore, Pakistan, over a period of 15 months from October 2019 to December 2020. The sample included diagnosed cases with first episode of haemorrhagic or ischemic stroke, of both genders, aged 40–60 years, having unilateral extremity involvement with a minimum score of 2 on medical research council scale. The unstable cases who could not follow instructions, cases with ischemic heart disease, unstable angina, history of seizers, motor impairments such as neuropathy or Parkinson's disease, aphasia, cognitive compromise that can interfere with comprehension of commands, and any systematic disease were excluded from the study. The participants were randomly assigned to virtual reality (*N* = 34) and routine physical therapy (*N* = 34) groups by the lottery method.

The current study was conducted after obtaining ethical approval of research from Institutional Research Board (IRB) of The University of Lahore vide Ref No. IRB-UOL-FAHS/373-III/2018 and registration of trial vide registration number RCT20190715044216N1 and after acquiring consent of participants. Consort guidelines were followed to screen participants for inclusion in the study (Figure 1).

The Berg balance scale (BBS) and Fugl-Meyer assessment tool for lower extremity (FMA-LE) were used for data collection. All the values were measured preintervention, immediate postintervention, and at 6 weeks postintervention. The period of 6 weeks was chosen to avoid patients being lost to longer follow-up.

The BBS is a valid and reliable tool to assess balance and functional mobility in stroke patients [25], and FMA-LE is a valid and reliable tool to measure function of lower extremity in the stroke patients [26].

The FMA comprises of 5 domains and 155 items analyzing motor and sensory function, balance, joint motion range, and joint pain and scored on 3-point scale, where O = cannot perform, 1 = partial performance, and 2 = full performance with maximum possible score being 226. BBS has 14 items scored 0–4 for 56 points with higher score indicating lower risk of falling.

Intervention with virtual reality training was instituted using Nintendo Wii home video game console [27], and the Nintendo Wii fit balance games were used. These require the patient to shift his/her weight while standing on the balance board. The overall intervention includes the following activities: (1) Wii balance games, e.g., tilt table and skiing, that target weight shifting in different directions, (2) Wii aerobics, e.g., stepping on balance board and running on spot, (3) Wii strength training includes Matt exercises and dynamic standing that targets weak muscles for strength, and (4) Wii yoga for static exercises. Balance board was put in the middle of parallel bars for any upper extremity assistance required by the patient in case of imbalance during exercise [28–30].

The article "A Novel Virtual Reality Training Strategy for Poststroke Patients: A Randomized Clinical Trial" was published in 2021. Journal: J Healthc Eng.

The patient played the game in real time natural environment and received 60-minute sessions four times a week for six weeks and training complexity and intensity changed according to patient's performance [27], while the PT group received 60-minute sessions, four times a week for six weeks including stretching exercises for tight muscles specially flexors in lower limb. The strengthening program is for weak extensor muscles and balance training, and coordination exercises is to improve motor control and deficit. Each muscle group was targeted for strengthening exercises in lower limb. Manual resistance was applied and increased according to the patient's condition. The motivational sessions included motivation of each patient by the researcher before and after each session for both groups to participate actively during the session.

The sampling technique used was convenience sampling using the online sample size calculator [31], with statistical power of 80% and *α* = 0.5. The total 76 participants were recruited to compensate dropout during the intervention.

The SPSS 22.0 was employed for statistical analysis. Descriptive statistics were applied for all outcome measures. Repeated measure ANOVA was used to compare between groups. Statistical significance was set at *p* < 0.05.

## 3. Results and Discussion

### 3.1. Results

The study population had a normal sample distribution with no significant difference between the VR and PT groups (Table 1).

Results revealed (Table 2) a statistically significant difference between the BBS score for the time main effect as well as time vs. group interaction (*p* < 0.001) with significantly higher scores indicating improved balance for the virtual reality group. There was a statistically significant difference in mean scores of FMA-motor function (FMA-MF), FMA-joint range (FMA-JR), and FMA-joint pain (FMA-JP) for both the time main effect and time vs. group interaction (*p* < 0.001) with significantly higher scores for virtual reality training indicting improved motor function, joint range, and pain. However, no significant difference was noted for FMA sensation (FMA-S) for time vs. group interaction (*p*=0.202); however, it was significant for the time main effect (*p* < 0.001).

The article "A Novel Virtual Reality Training Strategy for Poststroke Patients: A Randomized Clinical Trial" was published in 2021. Journal: J Healthc Eng.

### 3.2. Discussion

Virtual reality training is a modern technique of treatment receiving great attention because of being economical, and it provides motivation to the patient due to realistic visual objects and multiple sensory stimuli and the freedom of use, hence becoming more important for Pakistan due to the fact that stroke has revealed epidemiological and clinical picture which is in contrast to the Western literature with involvement of relatively younger population due to different risk factors [17, 18], and the need for economical strategies [16] being a developing economy with the weak healthcare system.

Schrodre et al. in their study concluded that VR is a good tool to increase patients' motivation towards rehabilitation and balance training, and the combined effects with other therapies enhance the patient's recovery [32]. It is significant for the present national stroke scenario that the current study revealed a significant difference for BBS score values (*p* < 0.001) with significantly higher scores of 36.62 ± 7.76 and 44.09 ± 9.37 for virtual reality compared to 26.94 ± 6.46 and 30.97 ± 7.48 for the physical therapy group indicating improved balance for the virtual reality group. Similarly, Kumar et al. reported that hemiplegic patients using Wii balance board performed weight shifting showed a significant difference in final catch trial [33]. Another study by Lee et al. reported improvement in specific outcomes for VR programs which showed most effective results of muscle strength, balance, joint range, gait, and muscle tension of lower limb and improve activities of daily living (ADL's) in stroke patients with the moderate effect [16]. Similar results, regarding improvement in balance, have been reported in the current study and in previous studies suggesting that VR is a beneficial tool to improve balance in the stroke population because patients enjoyed these games and spent more time with these gadgets and exercise repeatedly to show better performance, enhancing self-motivation, ultimately leading to increased number of repetitions and patient's retention and learning skills being considerably improved [32].

According to O'Briena et al., VR training in stroke population has significant impact since it improves patient's interest towards exercises with different gaming techniques and also increases repetitions with substantial impact on patient's condition. This technique activates the neurophysiological level, enhances neural activity, promotes excitability of cortical spinal level, and engages patient's ipsilateral and contralateral brain regions [34]. A local study by Salman reported that VR gaming was an effective treatment method to improve motor as well as sensory function indicating neuroplasticity in cases with hemiparesis following stroke and help the patient gain his/her functional ability [10]. Similarly, the present study revealed significantly higher (*p* < 0.001) scores for virtual reality training for FMA-motor function. These significant results are close to a RCT conducted by Vitor Antonio in 2019 which supports our study that the VR group is effective for motor functioning of the lower limb patients [35]. Another comparable study revealed greater influence on patient's movement restoration of the affected lower limb after stroke as compared to the other standard therapeutic interventions [11]. VR in contrast to prolonged, monotonous nature of PT raises patients interest by cutting down boredom and augments visuospatial feedback [10]; hence, it suits the Pakistani stroke population which is relatively younger [19].

The article "A Novel Virtual Reality Training Strategy for Poststroke Patients: A Randomized Clinical Trial" was published in 2021. Journal: J Healthc Eng.

In the present study, no significant association was noted in FMA-sensation for time vs. group interaction (*p*=0.202), while it was significant for the time main effect (*p* < 0.001). Carey et al. in a study conducted in 2016 stated that a literature gap exists in understanding how sensory function is achieved in stroke patients; therefore, further multidisciplinary approach and advancement as a prerequisite in field is necessitated [36].

The current study revealed significant improvement (*p* < 0.001) for FMA joint range with significantly higher scores for VR training. In positive correspondence to the current study, another international research by Lee et al. postulated that VR training is most effective in improving joint range of motion and kinematics, hence improving ADL's and the patient's Qol [16], while another study conducted by Junior VADS et al. also supported the current study that VR programs improve the movement of the lower limb which in turn augments mobility leading to functional independence with improved Qol [35].

The present study exhibited significant (*p* < 0.001) improvement of FMA pain scores with higher scores for virtual reality training. Similarly, Junior et al. reported significant results in improving pain scores in poststroke patients using VR [35], while a study conducted by Shahnaz suggested that nonimmersive VR is adjunct intervention in PT and can be recommended for the management of acute to chronic pain, since it works as a counterirritant and diverts the patient's attention from painful stimulus, thus decreasing the analgesic need and also improving the tolerance to painful stimuli [37].

The article "A Novel Virtual Reality Training Strategy for Poststroke Patients: A Randomized Clinical Trial" was published in 2021. Journal: J Healthc Eng.

The usefulness of the VT approach in treatment of poststroke cases is a useful strategy and the current study strengthens the role of virtual reality training in the treatment of poststroke balance and lower limb functional improvement with special reference to the 40–60 years age group.

## 4. Limitations

The current study was conducted in one centre of the country, and hence, results cannot be generalized therefore necessitating larger trials.

## 5. Conclusions

The current study concluded that virtual reality training proved more effective to restore balance and lower extremity function compared to conventional physical therapy in stroke patients though no significant difference in sensory improvement transpired. The present research has significant propositions for clinicians with better case management enhancing quality of life of patients along with the dearth of local literature, thus providing base for future research for a developing country.

## Figures and Tables

**Figure 1:** Methodology: consort flow diagram.

**Table 1:** Demographic characteristics (*N* = 68).

Variable	Virtual reality training group	Routine physical therapy group	*P* value
	Mean ± SD/*n*	Mean ± SD/*n*	
Age (years)	51.56 ± 7.19	51.35 ± 5.78	0.897
Weight (kg)	86.5 ± 11.41	86.35 ± 11.70	0.958
Height (meter)	1.68 ± 0.11	1.68 ± 0.09	1.000
Bone mass index (kg/m^2^)	30.66 ± 4.24	30.60 ± 4.67	0.057
Gender			
Male	20	14	0.146
Female	14	20	

**Table 2:** Pre and postintervention results for virtual reality and routine physical therapy treatment: RM-ANOVA statistics (*N* = 68).

Scale	Scale domain	Intervention timing	Training group		ANOVA statistics			
			Virtual reality	Routine physical therapy	Time main effect		Time ∗ group interaction	
			Mean ± SD	Mean ± SD	*F*	*P* value	*F*	*P* value
Berg balance scale		Preintervention	18.38 ± 5.19	19.68 ± 5.23	492.8	<0.001	77.8	<0.001
		Postintervention	36.62 ± 7.76	26.94 ± 6.46				
		Postintervention (6 weeks)	44.09 ± 9.37	30.97 ± 7.48				

Fugl-Meyer scale-lower extremity	Motor function	Preintervention	12.68 ± 3.67	13.74 ± 5.51	46.19	<0.001	52.37	<0.001
		Postintervention	26.38 ± 3.63	19.68 ± 4.96				
		Postintervention (6 weeks)	30.26 ± 3.12	22.76 ± 5.33				
	Sensation	Preintervention	9.91 ± 1.38	9.74 ± 1.54	73.7	<0.001	1.62	0.202
		Postintervention	10.76 ± 1.21	11.03 ± 1.14				
		Postintervention (6 weeks)	11.26 ± 1.02	11.30 ± 0.95				
	Joint range	Preintervention	10.47 ± 2.03	10.44 ± 2.03	423.68	<0.001	29.4	<0.001
		Postintervention	17.50 ± 1.11	14.18 ± 2.14				
		Postintervention (6 weeks)	19.03 ± 0.90	15.68 ± 2.22				
	Joint pain	Preintervention	11.50 ± 1.94	10.50 ± 1.99	472.69	<0.001	43.8	<0.001
		Postintervention	17.68 ± 1.51	13.50 ± 2.18				
		Postintervention (6 weeks)	18.97 ± 0.94	14.68 ± 1.90				

The article "A Novel Virtual Reality Training Strategy for Poststroke Patients: A Randomized Clinical Trial" was published in 2021. Journal: J Healthc Eng.

## Data Availability

The data used to support the findings of this study have not been made available because article is part of PhD research and will be available upon request after completion of degree program and defence from the corresponding author.
